# mtDNA structure: the women who formed the Brazilian Northeast

This article has been retracted.

**DOI:** 10.1186/s12862-017-1027-7

**Published:** 2017-08-09

**Authors:** Ana Paula Schaan, Lorenna Costa, Diego Santos, Antonio Modesto, Marcos Amador, Camile Lopes, Sílvia Helena Rabenhorst, Raquel Montenegro, Bruno D. A. Souza, Thayson Lopes, France Keiko Yoshioka, Giovanny Pinto, Vivian Silbiger, Ândrea Ribeiro-dos-Santos

**Affiliations:** 1 Human and Medical Genetics Laboratory, Federal University of Pará, Av. Augusto Corrêa, 01 – Cidade Universitária Prof. José Silveira Netto – Guamá, Belém, PA 66075-110 Brazil; 2 Clinical and Toxicological Analyses Department, Federal University of Rio Grande do Norte, Natal, RN 59300-000 Brazil; 3 Pathology and Legal Medicine Department, Federal University of Ceará, Fortaleza, CE 60020-181 Brazil; 4 Genetics and Molecular Biology Laboratory, Federal University of Piauí, Parnaíba, PI 64202-020 Brazil; 5 Center of Oncological Research, Federal University of Pará, Belém, PA 66073-005 Brazil; 6 Center of Research and Drug Development, Federal University of Ceará, Fortaleza, CE 60430-270 Brazil

**Keywords:** mtDNA lineages, Northeastern Brazil, Genetic diversity, Migration pattern, Population admixture, Asymmetric colonization

## Abstract

**Background:**

The distribution of mitochondrial DNA (mtDNA) lineages in Brazil is heterogeneous due to different regional colonization dynamics. Northeastern Brazil, although being an important region in terms of human imigration and ethnic admixture, has little information regarding its population mtDNA composition. Here, we determine which mitochondrial lineages contributed to the formation of the Northeastern Brazilian population. Our sample consisted of 767 individuals distributed as follows i) 550 individuals from eight Northeastern states (Piauí, Ceará, Rio Grande do Norte, Paraíba, Pernambuco, Alagoas, Sergipe, and Bahia) which were sequenced for mtDNA hypervariable segments I, II, and III; ii) 217 individuals from Alagoas and Pernambuco (previously published data). Data analysis was performed through sequence alignment and Haplogrep 2.0 haplogroup assignment tools. Furthermore, maternal ancestry distribution was contextualized and, when possible, related to historical events to better understand the biological interactions and population dynamics that occurred in this region since the beginning of colonization.

**Results:**

Unexpectedly, Amerindian mitochondrial ancestry was the highest in the Northeastern region overall, followed by African, European and non-Amerindian Asian, unlike previous results for this region. Alagoas and Pernambuco states, however, showed a larger African mtDNA frequency. The Northeastern region showed an intraregional heterogeneous distribution regarding ancestral groups, in which states/mesoregions located to the north had a prevalent Amerindian ancestral frequency and those to the south had predominance of African ancestry. Moreover, results showed great diversity of European haplogroups and the presence of non-Amerindian Asian haplogroups.

**Conclusions:**

Our findings are in disagreement with previous investigations that suggest African mitochondrial ancestry is the most prevalent in the Brazilian Northeast. The predominance of Amerindian lineages exemplifies the importance of indigenous women in the formation of the population, despite intense African slave entry and conflicts with European settlers. The variable distribution of ancestral groups observed in the Northeast is in accordance with historical records showing the similarities with colonization dynamics occurred in the Amazon region and the Brazilian Southeast. Moreover, the variety of European haplogroups suggests multiple origins of founding groups, specially those found in Western European populations.

**Electronic supplementary material:**

The online version of this article (doi:10.1186/s12862-017-1027-7) contains supplementary material, which is available to authorized users.

## Background

The Brazilian population is one of the world’s most ethnically diverse. This is the result of the colonization process of the territory by many different ancestral groups, including Amerindians, Europeans and Africans, over distinct time periods. Amerindians were the first settlers, immigrating to the American continent from eastern Asia between 11,000 and 25,000 years BP [1–5].

When the Portuguese came ashore at the Northeastern coast of Brazil in the 16th century, the native population was made up of an estimated 1–6.8 million individuals who spoke over 150 different languages, some of which were organized in complex sociopolitical systems [6, 7]. The European colonization involved military conflicts and the spread of diseases for which the natives had no natural defenses, resulting in great population decimation, and consequent loss of genetic and cultural diversity [7]. These groups were enslaved by the new settlers and forced to work in the extraction of Brazilwood, which was the first enterprise of the Portuguese crown in Brazilian territory [8, 9].

African slaves were later introduced to work at sugar cane plantations located mostly in the Northeastern region of Brazil. An estimated number of more than 700 thousand African individuals were forcibly brought to Brazil during the 16th and 17th centuries and by the 19th century, approximately 5 million Africans had arrived [10].

Occupation of the Brazilian territory intensified in the 17th century, especially in the Northeast. In the midst of the European competition for products, labor force, and markets, certain nations came to invade and dominate portions of the territory during the 16th and 17th century, including the French, English, and Dutch. This second wave of migrations possibly increased the genetic diversity in this region, as it was considered a strategic spot for colonization. The French attempted to settle in the Northeast in the late 1500s by invading the coast and, later, successfully occupied the Northeastern states of Maranhão, Paraíba, and Pernambuco, from which they were eventually ousted by the Portuguese [11, 12]. The English presence in Brazil during the first centuries of European colonization was limited to a small settlement on the Oiapoque river (located to the north) built in 1604; abandoned a year later [13]. In the 19th century, the English came to occupy the state of Pernambuco [14]. The Dutch invaded and dominated a significant portion of the Northeast territory in the 17th century; their settlements were then referred to as Brasil Holandês (Dutch Brazil) [15–17].

Due to the various processes involved in the formation of the Brazilian population, we must consider the incorporation of genetic markers from foreign colonizers and the historical processes that consequently introduced them. Thus, molecular biology is a well suited tool for tracing genetic markers left by this complex admixture process, for instance, through the investigation of maternal ancestry determined by the mitochondrial DNA (mtDNA) molecule. The control region of the mtDNA molecule is the most informative in terms of maternal ancestry and consists of three hypervariable regions (HVR-I, HVR-II and HVR-III), that collectively are capable of informing one’s ancestral haplogroup through the presence of specific motifs varying from a reference sequence [18, 19].

Little is known about the bioanthropological profile of the populations from Brazil’s Northeast region, despite its importance regarding population dynamics throughout history. Therefore, characterization of mtDNA genetic markers may clarify the colonization process that occurred in this region and complement previous knowledge on the biological composition of the Brazilian population. Here, we determine, through sequencing the entire control region, which lineages contributed to the formation of the Northeastern Brazilian population.

## Methods

### Population sample

Ethical consent was obtained according to the Helsinki Declaration. Ethical approval was obtained from the Research Ethics Committee of the Federal University of Rio Grande do Norte, Federal University of Piauí, and Federal University of Ceará, under protocol numbers 27,493,614.0.0000.5293, 0443.0.045.000–11, and 702/04, respectively. Before signing the Consent Form participants were informed regarding the nature of this research and use of their biological samples. All the analyses were performed preserving subjects anonymously throughout the study.

The sampled population (Fig. 1, Table 1) consisted of 767 non-related blood donor individuals from urban areas of Northeastern Brazil distributed as follows i) 550 individuals from eight northeastern states, from which (a) 174 represented the four mesoregions of Piauí state (North, Central-North, Southeast, and Southwest), (b) 52 from Fortaleza city, in the state of Ceará, (c) 276 from all four mesoregions of the state of Rio Grande do Norte (East, Agreste, Central, and West), (d) 21 from the state of Paraíba, (e) 14 from the state of Pernambuco, (f) two from Alagoas state, (g) four from the state of Sergipe, and (h) seven from the state of Bahia; ii) 50 individuals from Pernambuco state and 167 individuals from Alagoas state previously published in the literature [20, 21].

**Fig. 1:** Map of Northeastern Brazil with investigated areas, made up of eight states, highlighted in gray. (MA – Maranhão, PI – Piauí, CE – Ceará, RN – Rio Grande do Norte, PB – Paraíba, PE – Pernambuco, AL – Alagoas, SE – Sergipe, BA – Bahia)

**Table 1:** Investigated populations from Northeastern Brazil

Populations		Number	Reference
Piauí	North	45	Present study
	Central-North	42	
	Southeast	42	
	Southwest	45	
Total		174	
Ceará		52	Present study
Total			
Rio Grande do Norte	East	193	Present study
	Agreste	26	
	Central	29	
	West	28	
Total		276	
Paraíba		21	Present study
Total			
Pernambuco		64	Alves-Silva et al., 2000 [20]; present study
Total			
Alagoas		169	Barbosa et al., 2008 [21]; present study
Total			
Sergipe		04	Present study
Total			
Bahia		07	Present study
Total			
Total		767	-

### Genotyping

Biological material was obtained from a 5 mL peripheral blood sample from each individual, which was collected and stored in vacutainer tubes using EDTA as an anticoagulant. Later, DNA was extracted by the Sambrook et al. (1989) [22] method with modifications. The presence of mutations in the three hypervariable regions of the mtDNA control region were determined through conventional polymerase chain reaction (PCR) with primers L15997 (5′-CACCATTAGCACCCAAAGCT-3′) and H017 (5′-CCCGTGAGTGGTTAATAGGGT-3′) for HVR-I and L034 (5′ CCATGCATTTGGTATTTTCG-3′) and H629 (5′-TTTGTTTATGGGGTGATGTGA-3′) for HVRII/III. Thermocycling was performed using Vereti 96 Well equipment (Life Technologies, Foster City, CA-US) under conditions of initial denaturation at 95°C for 15 min followed by 35 cycles of denaturation at 95°C for 30 s, annealing at 60°C for 1 and a half minute and extension at 72°C for 1 min; final extension was at 72°C for 10 min. Amplification products were sequenced by automatic sequencer platform ABI 3130 (Life Technologies) in two separate reactions for each sample using the same PCR primers, aiming HVR-I with primer L15997 and HVR-II/III with L034. These analyses were carried out at the Medical and Genetics Laboratory in the Federal University of Pará (PA, Brazil).

### Data analysis

The resulting sequences were analysed by comparison with the revised Cambridge Reference sequence [18] using the National Center for Biotechnology Information (NCBI) database along with AMBASE software, produced by the UFPA Computational Biology Laboratory (unpublished data, available at lbcgh.ufpa.br/ambase). Haplogroups were determined with the help of Haplogrep 2 (v2.1.0) [23] and Phylotree (mtDNA tree Build 17) [19]. Individuals were then classified based on their mitochondrial ancestral origin, namely Amerindian, African, European, and non-Amerindian Asian. To evaluate the differences in the relative proportions of ancestral populations in the studied area, we performed Fischer’s exact test and ANOVA on R software (version 3.3.1) [24]. Diversity measures were computed on softwares MEGA7 [25] and DnaSP v.5.10.1 [26].

## Results

Overall, results showed that the population of the Northeastern region of Brazil has Amerindian mitochondrial ancestry as the most frequent, representing 43.5% of the individuals, followed by African (37.8%), European (16.6%), and non-Amerindian Asian (2.1%) (Table 2). Individually, Amerindian ancestry was also the most prevalent in five out of eight investigated states from Northeastern Brazil (Piauí, Ceará, Rio Grande do Norte, Sergipe, and Bahia), followed by African, European and Non-Amerindian Asian. The states of Pernambuco and Alagoas presented African mtDNA ancestry as the most frequent while Paraíba revealed the same frequencies for Amerindian and African mitochondrial lineages; these states also presented European haplogroups as the least frequent ancestral groups. Due to small sample size representation, we chose to exclude the states of Sergipe and Bahia from further analyses.

**Table 2:** Ancestral group frequencies among investigated states. AMR – Amerindian, AFR – African, EUR – European, ASI – Non-Amerindian Asian

Populations		Number	Frequency (%)			
			AMR (N)	AFR (N)	EUR (N)	ASI (N)
Piauí	North	45	51 (23)	31 (14)	11 (05)	7 (03)
	Central-North	42	69 (29)	24 (10)	7 (03)	-
	Southeast	42	39 (17)	43.9 (18)	17.1 (07)	-
	Southwest	45	48.9 (22)	46.7 (21)	4.4 (02)	-
Total		174	52.3 (91)	36.2 (63)	9.8 (17)	1.7 (03)
Ceará		52	51.9 (27)	30.8 (16)	11.5 (06)	5.8 (03)
Rio Grande do Norte	East	193	45.6 (88)	35.8 (69)	15.5 (30)	3.1 (06)
	Agreste	26	50 (13)	34.6 (09)	11.5 (03)	3.8 (01)
	Central	29	44.8 (13)	20.7 (06)	24.1 (07)	10.3 (03)
	West	28	42.9 (12)	46.4 (13)	10.7 (03)	-
Total		276	45.7 (126)	35.1 (97)	15.6 (43)	3.6 (10)
Paraíba		21	38.1 (8)	38.1 (08)	23.8 (05)	-
Pernambuco		64	30.3 (18)	40.8 (26)	28.9 (20)	-
Alagoas		169	33.1 (56)	45.6 (77)	21.3 (36)	-
Sergipe		4	75 (03)	25 (01)	-	-
Bahia		7	71.4 (05)	28.6 (02)	-	-
Total		767	43.5 (334)	37.8 (290)	16.6 (127)	2.1 (16)

In the state of Piauí, individuals descending from Amerindian maternal lineages accounted for 52.3%, followed by African, European, and non-Amerindian Asian, each with 36.2%, 9.8% and 1.7%, respectively. In Ceará, Amerindian lineages were present in 51.9% of the samples, followed by 30.8% African, 11.5% European, and 5.8% non-Amerindian Asian. Similarly, in Rio Grande do Norte 45.7% of the population has Amerindian ancestry, while 35.1% as African descendants, 15.6% are European and 3.6% are non-Amerindian Asian.

As mentioned above, Pernambuco had African mtDNA ancestry as the most frequent, present in 40.8% of the individuals, followed by Amerindian, 30.3%, and European, 28.9%. Likewise, African ancestry represented 45.6% of individuals in Alagoas, while Amerindians and Europeans corresponded to 33.1% and 21.3%, respectively.

After excluding Sergipe and Bahia from the analysis, Amerindian mtDNA ancestry continued to be the most frequent in the Northeastern region overall, with 43.1% of the population, while Africans corresponded to 38%, Europeans to 16.8%, and Non-Amerindian Asians to 2.1%.

Maternal ancestral group frequencies were further compared at the mesoregion level in the states of Piauí and Rio Grande do Norte. As a result, Piauí presented the following heterogeneous distribution (Fig. 2). In its Northern mesoregions (North and Central-North), Amerindian ancestry is prevalent at 59.8%, while Africans represent only 27.6% of the individuals, Europeans 9.2%, and Non-Amerindian Asians 3.4%. In the Southern mesoregions (Southeast and Southwest) we observed African ancestry as great as Amerindian, both contributing at 44.8% of the population; Europeans correspond to 10.8%. Fischer’s exact test was performed in 2 × 2 contingency tables to verify the presence of significant proportional differences and identified they are significantly different regarding the contribution of African descendants (*p* < 0.05).

**Fig. 2:** Heterogeneous distribution of mitochondrial ancestral groups in Piauí. Amerindian presence is prevalent to the North, while African and Amerindian ancestry are equally represented to the South. The frequency of European descendants is similar in both regions; non-Amerindian Asians are only found to the North

In Rio Grande do Norte, significant differences were not observed when considering the distribution of maternal ancestral groups among its mesoregions.

Among the Amerindian mtDNA haplogroups identified in our sample, haplogroup A was the most frequent, representing 34.7% of individuals with Native American ancestry. The most frequent African haplogroup, L3, was present in 38.2% of African descendants, with 61.1% of them belonging to sub-haplogroup L3e. The diversity of European haplogroups was larger than expected, although haplogroup H was the most frequent (*n* = 72), accounting for 56.7% of individuals with European ancestry. Additionally, haplogroups J (*N* = 10), HV (*N* = 6), K (*N* = 8), U (*N* = 13), T (*N* = 9), I (*N* = 1), JT (*N* = 1), W (*N* = 1), Pre-V (*N* = 1), and V (*N* = 3) were also present. Regarding non-Amerindian Asians, we identified haplogroups M (*N* = 8), N (*N* = 5), S (*N* = 2), and G (*N* = 1). This data is represented in Table 3 and Fig. 3. Figure 4 presents mtDNA haplogroup distribution per investigate population.

**Table 3:** mtDNA haplogroup frequencies per investigated state

Haplogroups	Frequency per Population (%)					
	Piauí (*N* = 174)	Ceará (*N* = 52)	Rio Grande do Norte (*N* = 276)	Paraíba (*N* = 21)	Pernambuco (*N* = 64)	Alagoas (*N* = 169)
A	23.6	13.5	13.4	4.8	14.1	10.7
B	9.2	13.5	15.2	19.0	7.8	10.1
C	12.6	21.2	13.0	9.5	1.6	10.1
D	6.9	3.8	3.6	4.8	4.7	2.4
X	-	-	0.4	-	-	-
L0	2.9	3.8	4.3	9.5	-	-
L1	9.2	9.6	4.3	4.8	14.1	14.8
L2	10.9	7.7	12.7	9.5	7.8	11.8
L3	13.2	9.6	13.4	14.3	18.8	16.6
L5	-	-	0.4	-	-	-
H	4.6	7.7	9.1	19.0	20.3	10.7
V	-	-	-	-	1.6	1.2
HV	1.7	-	1.1	-	-	-
Pre-V	-	-	-	-	-	0.6
I	0.6	-	-	-	-	-
JT	0.6	-	-	-	-	-
J	-	-	2.5	-	1.6	1.2
K	0.6	-	1.1	-	3.1	-
T	0.6	-	0.7	4.8	1.6	2.4
U	1.1	-	0.7	-	3.1	4.1
W	-	-	0.4	-	-	1.2
G	0.6	-	-	-	-	-
N	0.6	1.9	1.1	-	-	-
S	0.6	-	0.4	-	-	-
M	-	3.8	2.2	-	-	-
?	-	-	-	-	-	2.4
Total	100.0	100.0	100.0	100.0	100.0	100.0

**Fig. 3:** Distribution of mtDNA haplogroups in Northeastern Brazil. Amerindian haplogroups in shades of *green*; Non-Amerindian Asian haplogroups in shades of *gray*; African haplogroups in shades of *orange*; European haplogroups in shades of *blue*

**Fig. 4:** Distribution of mtDNA haplogroups in Northeastern Brazil distributed according to each investigated state. Amerindian haplogroups in shades of *green*; Non-Amerindian Asian haplogroups in shades of *gray*; African haplogroups in shades of *orange*; European haplogroups in shades of *blue*

Finally, the 550 samples processed in the present study generated a total of 447 unique mtDNA sequences considering all three hypervariable regions, with a mean resolution level of 87.7%. Other diversity measures are displayed in Table 4.

**Table 4:** Dversity measures estimated from the analysis of the entire mtDNA HVI + II + III regions in the population sample from Northeastern Brazil

Parameters	HV-I + II + III
Number of haplotypes	447
Number of polymorfic sites	210
Transition/Transversion Bias	6.91
Mean number of pairwise differences	11.041
Nucleotide diversity	0.1006
Haplotype (gene) diversity	0.998 ± 0.0004

## Discussion

The heterogeneous distribution of maternal lineages in Brazil has been previously demonstrated, given the diverse distribution pattern of maternal ancestral groups throughout the territory, [20, 21, 27–35] [see Additional file 1] and is expected due to multiple colonization processes across each geopolitical region. The predominance of Amerindian ancestry observed in this study (43.5%) demonstrates the importance of Native American groups towards the formation of Brazil’s Northeastern population. Moreover, our results for Piauí, Ceará, and Rio Grande do Norte, in which Amerindian ancestry is more frequent, can be compared to those found for the Northern population (59.2% of Amerindian mtDNA) [28–30]. Therefore, our findings do not corroborate the usual association between Northeastern Brazil and predominance of African maternal ancestry [20, 21].

However, results for Pernambuco and Alagoas are in agreement for what has been previously described, showing African ancestry is the most frequent in both states [20, 21], much like the Brazilian Southeast region [20, 30–32].

Overall, the population of the Northeast has a larger contribution of Amerindian mitochondrial lineages than that of Africans. This constitutes a remarkable presence and resistance of the Native American component considering the centuries of drastic population decimation through conflicts, ensalvement, and diseases. Also, the Northeastern region was the main port of entry for enslaved Africans, being that Maranhão, Pernambuco, Bahia, and Rio de Janeiro were the leading states for the arrival of slave ships (only the latter is not part of the Northeastern region) [11, 12, 36]. Thus, Native American maternal lineages constitute the majority despite intense African presence. This demonstrates that indigenous females have been more expressively incorporated to the genepool than African females. Also, this may be the result of indigenous demographic expansion occurred during the 20th century [37].

The unequal distribution of African and Native American lineages across the mesoregions of the state of Piauí seems to be due to colonization dynamics occurred during the 17th and 18th century. In fear of losing the land to foreign invaders and looking to expand subsistence activities, Portuguese settlers from the coast expanded inland in search of lands for raising cattle. Starting from the current states of Pernambuco and Bahia (located at the coast), they reached territories that are now in the state of Piauí and the western part of Maranhão. Cattle ranches were usually located along the rivers that drain to the south and southeast of Piauí [11, 38].

Economic expansion to the west led to great conflicts with indigenous groups, which again resulted in a decreased number of native peoples due to enslavement, escape, and death [39]. Thus, occupying the southern half of Piauí increased the presence of African slaves, who came from the coast to work at the ranches. The slave trade was also intense in this area considering the geographical location of Piauí, being in between the states of Maranhão and Pernambuco, which, as previously mentioned, were African slave arrival points [39].

Interpreting our results, we propose that the mtDNA lineage distribution in Northeastern Brazil be understood as a split into two different sets that follow regional colonization patterns (Fig. 5). The first includes states and/or regions with great Amerindian influence, in which the majority of the population has Native American ancestry, which is in accordance with previous results from the Amazon region [20, 27, 28]; the second includes states and/or regions with a significant African contribution, following the patterns found for Southeastern Brazil [20, 30–32]. This proposition is reinforced by the heterogeneous manner in which the population ancestry from Piauí is distributed and by the frequencies found for Paraíba, that show a general tendency towards an equilibrium between Amerindian and African descendants.

**Fig. 5:** Northeast Brazil divided into two sets regarding mtDNA ancestry. The variability in mtDNA composition seems to be related to European colonization events. The state of Paraíba, located in between both groups, showed equal frequencies for Amerindians and Africans and is, therefore, a transition between both sets

Individuals who were assigned non-Amerindian Asian mtDNA lineages in our results are most likely of East Asian ancestral background. Asian imigration to Brazil began in the 20th century with populations arriving specially from East Asian countries, such as Japan, who’s imigrants reached an estimated 200 thousand individuals by 1941 [40]. The most recent demographic census revealed that the population of Asian origin registered a growth of 176.4% from 2000 to 2010 (from other countries as well, such as Korea and China), specially in the Southeast and Northeast regions of Brazil [41, 42]. Thus, the Asian mtDNA haplogroups identified in our study are most likely from East Asian, as has been registered in previous studies [43, 44].

Haplogroups found in this study have also been mentioned in other publications regarding the Brazilian genepool. Concerning the African lineages observed in the present sample, the most frequent contribution of haplogroup L3e is consistent with findings from previous studies from the Northeast and other regions of Brazil [20, 21, 30–32]. Moreover, this is compatible with historical records, since L3e is known to have high frequencies in West-Central Africa, which was the main source of African slaves brought to Brazil during the colonial period [10, 45, 46]. Additionally, Amerindian haplogroup A has already been demonstrated to be the most frequent in the Northeastern region by Alves-Silva et al. (2000) and Barbosa et al. (2008) [20, 21].

Regarding the European component, the prevalence of haplogroup H is in agreement with previous descriptions of European lineages in Brazil [20, 21, 30, 32–35]. Nonetheless, the diversity of haplogroups observed displays the multiple origins of the settlers, highlighting mainly Western European populations [47–49]. The European lineage diversity found for Northeastern individuals has been shown also in male lineages, demonstrating Eastern European influx larger than the observed for other regions of the country [50].

When considering male uniparental markers, European lineages are the most frequent throughout the country, including the Northeastern region. The least frequent ancestral group is Amerindian [50–52]. Thus, this indicates strong directional mating, a common occurrence during the colonial period, in which European men were encouraged to mate with Indigenous and African females [11, 12], leading to differences regarding ancestral group frequencies in uniparental markers. Moreover, the sex biased mode of population composition has been described in other South American countries as well [53–56].

Regarding the obtained diversity measures, our results differed from those described in earlier studies from the Northeastern [21, 57] and Southern regions [34, 35], specially nucleotide diversity. However, our data was comparable to that previously described for the Southeastern population of Brazil [30, 32], which is characterized as being the major urban center of the country. This exemplifies that our data, derived from multiple Northeastern states, has similar diversity measures probably due to both regions being of intense gene flow associated with many migratory events.

## Conclusions

Technological improvements currently allow sequencing technologies, such as whole genome sequencing, to answer many questions regarding evolutionary genetics and large-scale population genomics, which may cause mtDNA control region sequencing data to be perceived as out-of-date. It is necessary to acknowledge that maternal lineage assignment alone does not provide a comprehensive overview of the ancestral profile of the targeted population. To do so, it is necessary to investigate Y chromosome lineages and genomic DNA as well. However, in largely admixed populations, it is important to analyse this uniparental profile in order to characterize its fundamental formation, which can also lead to cultural inferences. Therefore, mtDNA sequecing continues to be relevant for investigating population structure in complex populations, such as the one presented here, as well as for forensic purposes. In order to identify specific sex-related biases and other migration dynamics that may lead to unique population composition we must consider the mtDNA sequencing approach as capable of yielding valuable insights.

Our results show a previously unseen prevalence of Amerindian mitochondrial lineages in Northeastern Brazil despite centuries of Indigenous genocide and posterior miscigenation. Therefore, while the current Brazilian population has and continues to incorporate foreign genetic markers, the Native American mitochondrial DNA still predominates in the population. This demonstrates Indigenous women were essential to the formation of the Northeastern population to the extent that they are present in the majority of current individuals despite having been at the basis of the social period since European colonization events. The presence of multiple European haplogroups suggests the many origins of founding populations, specially from historical but also recent events of migration. Finally, the detection of non-Amerindian Asian haplogroups is a probable demonstration of recent Asian migratory waves that now begin to appear in a larger portion of the population.

## Additional file

Additional file 1: Mitochondrial DNA ancestral group frequencies in other Brazilian geopolitical regions. (DOCX 30 kb)

## Abbreviations

mtDNA: Mitochondrial DNA
